# Music Individualization Recommendation System Based on Big Data Analysis

**DOI:** 10.1155/2022/7646000

**Published:** 2022-07-05

**Authors:** Pengfei Sun

**Affiliations:** The School of Arts, Yangtze University, Jingzhou 434023, China

## Abstract

This study discovers a certain complementary relationship between different algorithms after conducting a comprehensive and in-depth analysis of proposal algorithms. This study proposes a big data music individualization proposal method based on big data analysis, which integrates user behaviour, behaviour context, user information, and music work information, based on traditional music proposal methods; improves the collaborative filtering proposal algorithm based on user behaviour; and calculates the semantic similarity between lyrics, as well as the song co-occurrence similarity based on the user's music download history. Because the lyrics represent the thoughts and feelings that the song wishes to convey to the listeners, the proposal module is completed, and the music proposal system is realized, by combining the two different similar information, using the improved algorithm and the Hadoop distributed framework. The music similarity and label similarity are combined to alleviate the problem of cold start and data sparseness, and a mixed similarity calculation formula is proposed to calculate the similarity between music. The accuracy similarity of the big data music proposal model proposed in this study is improved by about 20% through experimental comparison when compared with the collaborative filtering model and the hybrid model. It reflects the efficiency, scalability, and stability of the music proposal system as well as the ability to meet users' individual music needs.

## 1. Introduction

With the development of network technology, the music recommendation system has also developed rapidly, and online music platforms have become the first choice for people to listen to music. However, the music recommendation system also faces some problems, such as data storage confusion, low computational efficiency, cold start, and data sparsity caused by the large scale of data [1]. Aiming at the above problems, this study designs and implements a music recommendation system. Firstly, two channels of offline data transmission and real-time data transmission are designed to collect and transmit data. A music data warehouse is built to process and store the data in layers. Then the data are preprocessed to facilitate the calculation of the recommendation model [2]. Secondly, based on the improved algorithm, combined with the Hadoop distributed framework, the proposal module is completed, and the music proposal system is realized. Finally, after the functional test and nonfunctional test, it reflects the efficiency, scalability, and stability of the music recommendation system, which can meet the individualization music needs of users.

The core algorithm of the personalized music recommendation system developed in this article is the semantic-enhanced big data technology. Experiments show that when recommending unpopular music, the big data recommendation algorithm proposed in this article is more effective than pure content-based and collaboration-based recommendation methods. In order to meet the needs of the current huge user group to recommend massive music, the current mainstream big data distributed computing platform is used in the development of this system. Through a comprehensive and in-depth analysis of the two types of recommendation algorithms, it is found that there is a certain complementary relationship between the two types of algorithms. Therefore, this study proposes a semantic-enhanced big data technology [3] that combines content-based recommendation algorithms and collaborative filtering recommendation algorithms. The algorithm first analyzes the semantic information implied in the lyrics and calculates the semantic similarity between song lyrics, and then calculates the co-occurrence similarity of songs based on the user's music download history. Because the lyrics represent the thoughts and feelings that a song wants to convey to the listeners, this recommendation algorithm can improve the shortcomings of big data technology by combining these two different similar information [4]. The research object of this study is lyric songs. In the following, music and song refer to a song with lyrics.

Through the mapping relationship between interest degree and time, the algorithm introduces the influence of time decay factor when calculating the item rating matrix through historical behaviour, so as to obtain a more accurate recommendation result [5]. In the face of the cold start problem, a hybrid recommendation mode based on tags and collaborative filtering is adopted. When the system is first deployed and the number of users and rating items is less than a certain threshold, the songs are matched by the initial preference tag when the user registers, whereas when the number of users is sufficient, the improved collaborative filtering algorithm is used for music recommendation. The user's operations are monitored and recorded in real time, and the user's personalized recommendation list will be updated accordingly. The system should be developed by investigating the needs of users, referring to the current excellent music recommendation system, designing each functional module of the system, developing a good user interface, and aiming to design an accurate and easy-to-use system of personalized music recommendation [6].

The innovation of this study are as follows: the proposal algorithm combined with user behaviour analysis realizes the proposal according to a series of user behaviour records. The model, according to the complexity and diversity of user interests, learns the influence of different attributes on user interests.

The rest of the article is organized as follows: Section 2 introduces related big data technology concepts. Section 3 applies big data technology to the individualization music model. Section 4 applies big data technology [7] to the individualization music model. Based on the proposed big data proposal model, collaborative filtering model, and hybrid model, the section makes recommendations. Section 5 summarizes the entire article.

## 2. Related Works

Common recommendation methods have a number of flaws, including the inability to improve recommendation effects, migrate with changes in users' hobbies, mine users' potential hobbies, and make accurate recommendations based on users' hobbies. However, with the rapid development of big data and artificial intelligence [7, 8], traditional recommendation methods can now be improved. To meet users' daily needs, we can combine the benefits and drawbacks of traditional recommendation methods with new elements, as well as learn from each other. As a result of the new circumstance, the music recommendation system should also keep up with the pace of change. It is critical at this time to design and implement a comprehensive music recommendation system that is both accurate and easy to use. It is critical to create a music recommendation system that provides a better user experience.

Wang et al. implemented a user-based collaborative filtering algorithm on the cloud computing platform Hadoop, which solved the scalability problem of the collaborative filtering algorithm [9]. Yuqiao et al. used a collaborative filtering proposal algorithm to use user preference data to predict products that new users may like [10]. Hu et al. introduced matrix factorization techniques applied in recommendation systems and analyzed the impact of each matrix factorization technique on recommendation systems [11]. Tong et al. studied a hybrid proposal algorithm based on collaborative filtering and used the dimensionality reduction method of singular value decomposition to find the most similar items and users in item clusters and user clusters, which effectively improved collaboration [12]. Zhang et al. proposed a collaborative filtering proposal algorithm based on the social network. Based on the traditional matrix factorization model, the user preferences of social networks were integrated to obtain a trust feature matrix, which reduced the impact of data sparsity [13]. Liang et al. proposed a new deep learning model to utilize image content for content proposal in social networks. W. Cai et al. [7] applied the k-means clustering algorithm to a traditional content-based proposal and proposed a new proposal algorithm [14]. Chen et al. proposed the field of music proposal. The previous collaborative proposal can no longer meet the requirements of the audience. The essence of music proposal has become the proposal of listening experience. The article describes the solutions to the current music proposal problem in academia and industry: playlist generation, contextual proposal, and music production proposal [15]. Huang et al. proposed research on the robustness of recommender systems, including classifying the types of proposal model attacks, computing the impact of research attacks, and recommending replacement plans [16]. Jiang et al. reviewed and summarized the principles and challenges of recommender systems used in online music and looked forward to some future techniques that might be used to improve music proposal results [17]. Zhang et al. believed that traditional proposal systems try to help users find related items, but this is not enough. Proposals need to give more appropriate results based on the time and location of the user at that time, that is, considering the scene recommended [18]. Bauer and Schedl first extracted acoustic features from the audio inquiries and used the content-based collaborative filtering proposal method to complete music proposal. Domestic scholars' research on music individualization proposal has also formed a series of scientific research results [19]. Su et al. used spectrogram analysis to obtain the characteristic data matrix of musical works and calculated the similarity between stored music and query data to achieve Top-N proposal [20]. Zhang et al. studied the multi-domain recommender systems, because traditional recommender systems only consider items in the same field, while cross-field recommender systems support operations on items in different fields, making the recommender system more accurate [21]. Feng used the method of bibliographical analysis to complete the proposal algorithm from different perspectives by using differential strategies and analyzed various descriptions of music-related documents to obtain its regularity to complete the proposal [22].

In this era of excess data, there are various connections between data, and it is obviously unrealistic to rely on humans to distinguish. However, with the rise of big data technology, various tools for data processing have made it possible for us to discover the internal connection of data. This is a significant breakthrough by mining potential connections between data and serving recommender systems. Data can be analyzed from multiple perspectives, such as user behaviour context, scene atmosphere, time perception, etc., to improve the accuracy of the proposal system from multiple perspectives.

## 3. Concepts Related to Individualization Proposal Technology Based on Big Data Analysis Technology

Data acquisition is the basic premise of processing. With the rapid development of the Internet, Internet of Things, and cloud computing, they have become important channels for obtaining data. Especially with the rapid development of smart mobile terminals, a large amount of data is generated every day, among which mobile phones and mobile terminals are representative.

The main functions of data integration are data extraction, cleaning, and storage. The data collected during the data acquisition stage are typically large in scale and diverse in nature. Data extraction's main goal is to convert complex data types into unified or easy-to-understand data structures. The amount of data collected is usually large, but the amount of valid data is not. Many of the data may be of little or no use in specific application scenarios, and even more data may contain incorrect information. Data cleaning ensures data quality, while data storage serves as a platform for data processing. The core of the processing process and the process of extracting useful information from big data is data analysis. The only way to get useful information is to use the right method. After the user's historical data, such as search terms, have been used, it is saved in the database and never used again. Big data typically contain some basic data, and valuable information can be mined by expanding these data. Parts of the data have less value than the overall value, so different data sets are reorganized for analysis to achieve a relatively high total value. Sometimes useful information can be found in error data, such as spell-checking during searches. The Internet can be used to obtain very public data, and the majority of them are obtained by advanced enterprises and research institutions both at home and abroad. These open data can be used by researchers to conduct research and create more value. The user is presented with the processed results during data interpretation. In contrast to data analysis, which requires professional knowledge, the results of data processing are displayed to ordinary users who do not necessarily understand the technology of data analysis. As a result, how to clearly display the results to ordinary users is a critical issue, which is usually accomplished through the use of graphics, charts, or tabular methods.

As shown in Figure 1, user 1 purchases three items A, B, and D, and user 3 purchases items B and D. By analyzing the purchase behaviour of users, it can be found that the similarity between user 1 and user 3 is relatively high. Among them, user 1 has purchased item A, so it can be inferred that user 3 is very inclined to purchase item A, so it is recommended to user 3.

The concept of big data technology has been deeply influenced at the interaction level. This chapter will combine the theory of interaction to expound the interaction in music. Audience research has become an increasingly important part of social media research. When the real interpersonal communication is more and more carried out in the virtual network, the social activities between people will also change more or less, which are shown in Figure 2.

The algorithm is divided into three steps: the first is item representation, in which we must extract the item's content features to represent the item; the second is song recommendation, in which we can use the song's tags as well as the singer's tag and other features; and the third is item recommendation, in which we must extract the item's content features to represent the item. We can use the user's historical behaviour to describe the user's item feature preference for feature learning. This type of preference can be expressed in music recommendations based on the user's song behaviour data. Finally, a recommendation sequence is generated, and through similarity comparison, a set of items with the highest similarity is generated for the user. Data on the user's online behaviour are collected and stored. User online behaviour refers to a user's new behaviour, such as listening to new songs, dancing to new songs, collecting albums, saving the data in the appropriate database, and classifying the information in the database. Users can sort their preferences, and they can check their listening records at any time. When a user contacts the system and registers as a new user, the user can display the music he likes and hide the music he does not like based on his personal preferences, and the user can change the information set by himself at any time. The music recommendation system can recommend songs that the user is interested in and prevent songs that the user does not like from appearing in his music playlist based on the user's music preference information.

## 4. Design of Music Proposal Model Based on Big Data Analysis

### 4.1. User Preferences Similarity Calculation Based on Big Data Analysis

The similarity formula is used at the heart of massive data technology to calculate project similarity, and the similarity that can be selected for different projects is also different. Massive data technology, in comparison to collaborative filtering and mixed model algorithms, can learn the influence weights of different attributes and the interaction between attributes on user interests. Big data technology, for example, can learn not only the impact of a single attribute on user interest, but also the impact of any combination of attributes. Using the example of user age, gender, and time, big data technology can determine the impact of these three attributes alone on user interest as well as the impact of any two or even three attributes combined on user interest. This is classic modelling. Algorithms are incapable of accomplishing this. This study takes into account the impact of modelling and the amount of computation, but only considers the impact of a single attribute and any two attributes on user interest.

The user information is represented as *X*(*x*)={*x*1, *x*2, ..., *xz*, *y*} after processing, where *y* is the user's preference value for the item expressed by this behaviour, and *xi* is the value of the *i* feature of the user's current behaviour. The method of big data technology is to use user data to pass learning to obtain a prediction function *f*(*x*). It represents different interest models of users, and the calculation formula is as follows:

(1) $$\begin{array}{c} f\left(X\right)=w_{0}+\sum_{i=1}^{n}w_{i}x_{i}+\sum_{i=1}^{n}\sum_{j=i+1}^{n}v_{ij}x_{i}x_{j}, \end{array}$$

where *w*_0_ is the global parameter deviation, *x*_*i*_ is the value of the *i* attribute of the user's current behaviour, the meaning of the *w*_*i*_*x*_*i*_ part is the contribution of the attribute *x*_*i*_ to the user's interest, and *v*_*ij*_*w*_*i*_*x*_*j*_ represents the effect of the attributes *x*_*i*_ and *x*_*j*_ on the user's interest.

The data set is to learn the function *f*(*x*) by using big data technology on the data in the data set. The purpose of the test set is to test the learning effect of the function *f*(*x*). The following formula defines the loss function *L* of the big data technology:

(2) $$\begin{array}{c} L=\sum_{i=1}^{N}\text{loss}\left(f\left(X\right),Y\right)=\sum_{i=1}^{N}{\left(\hat{y}\left(x_{i}\right)-y_{i}\right)}^{2}. \end{array}$$

In the pursuit of minimizing the loss function, it is necessary to prevent the occurrence of overfitting. The regularization term in this article introduces the parameter vector formula (3), which is the calculation of the optimization problem of big data technology.

(3) $$\begin{array}{c} L=\arg\min\sum_{i=1}^{N}{\left(\hat{y}\left(x_{i}\right)-y_{i}\right)}^{2}. \end{array}$$

The above formula represents all the model parameters of big data technology, that is, the specific influence weights of attributes on user interests. There are two related functions *g*(*x*) and *h*(*x*) for any parameter of *f*(*x*), as shown in the following formula:

(4) $$\begin{array}{c} \hat{y}\left(x\right)=g\left(x\right)+h\left(x\right). \end{array}$$

When *w*_0_=0,

(5) $$\begin{array}{c} \hat{y}\left(X\right)=\sum_{i=1}^{n}w_{i}x_{i}+\sum_{i=1}^{n-1}\sum_{j=i+1}^{n}\left(v_{i}^{T}v_{j}\right)x_{i}x_{j}+w_{0}. \end{array}$$

When *w*_0_=1,2, ..., *n*, as shown in (5),

(6) $$\begin{array}{c} \hat{y}\left(x\right)=w_{0}+\sum_{i=1}^{n}w_{i}x_{i}+\sum_{i=1}^{n-1}\sum_{j=i+1}^{n}\left(\sum v_{ls}v_{js}\right)x_{i}x_{j}. \end{array}$$

Only one parameter is optimized in each calculation process, and the iterations are performed round by round. Music can usually have a variety of tag information, which can be analyzed and described from different dimensions. The more tags, the better the representation of items. Each piece of music has a different label, and the more common labels between two pieces of music, the more similar they are. The calculation formula for defining the similarity of labels is as follows:

(7) $$\begin{array}{c} {\text{sim}}_{tah\left(u,v\right)}=\frac{I_{u}\cap I_{v}}{I_{u}\cup I_{v}}. \end{array}$$

The tag-based proposal algorithm can still recommend music in the absence of user ratings and alleviate the problem of cold start to a certain extent. Although the tag-based proposal algorithm does not require the user's score record, only the tag of the music itself is needed. Combining the tag-based proposal algorithm with other proposal algorithms can improve the proposal effect.

### 4.2. Music Score Clustering Algorithm

Each user has his own scale when scoring the music. For a very favorite item, conservative-type users rate lower than positive-type users. From a mathematical point of view, different users have different mean and variance of ratings. Therefore, in order to have a unified standard for user preferences, it is necessary to normalize user ratings. In the method based on the clustering algorithm, the principle is to subtract the average of the user's score from the user's score on the music, which is shown in the following formula:

(8) $$\begin{array}{c} h\left(r_{ui}\right)=r_{ui}-{\bar{r}}_{u}. \end{array}$$

Bringing formula (8) into formula (9), we can get the predicted user *u* score for the new music *i* as

(9) $$\begin{array}{c} r_{ui}={\bar{r}}_{u}+\frac{\sum_{v\in N_{i}\left(u\right)}w_{uv}\left(r_{vi}-{\bar{r}}_{v}\right)}{\sum_{v\in N_{i}\left(u\right)}\left|w_{uv}\right|\sum_{}} \end{array}$$

The special feature of big data technology is that normalization takes into account the variance of user ratings. For user-based methods, the definitions are shown in the following expression:

(10) $$\begin{array}{c} h\left(r_{ui}\right)=\frac{r_{ui}-{\bar{r}}_{u}}{\sigma_{u}}. \end{array}$$

Bringing this formula into formula (9), the user's rating of the new music can be predicted, which is shown in the following formula:

(11) $$\begin{array}{c} {\overset{⌢}{r}}_{ui}={\bar{r}}_{u}+\sigma_{i}\frac{\sum_{j\in N_{i}\left(i\right)}\left(w_{ij}\left(r_{vj}-{\bar{r}}_{j}\right)/\sigma_{j}\right)}{\sum_{j\in N_{i}\left(u\right)}\left|w_{uv}\right|}. \end{array}$$

### 4.3. Individualization Proposal Model Based on Big Data Technology

The main component of the recommendation module is the recommendation model, which is the heart of the recommendation system. As a result, the user experience is directly related to a good recommendation model. After analyzing and summarizing a variety of common recommendation models, it was discovered that each model has distinct advantages and disadvantages in terms of generating an accurate user recommendation list. This system uses a hybrid recommendation system that relies heavily on the use of tags and collaborative filtering. When the number of users or the number of user-rated items is insufficient, a tag-based recommendation model is used. This is primarily used to address the collaborative filtering recommendation problem—problem with cold start. The improved collaborative filtering algorithm is enabled when the number of users and user rating items is sufficient. Time considerations are introduced into traditional collaborative filtering because users' interests may change over time.  Figure 3 depicts the recommendation process for accurate recommendations.

The core idea behind the big data-based recommendation algorithm is to use audio features to describe a piece of audio data, and then use those features to calculate similarity with other audios. It analyses the feature information of the tracks, traverses the music database, and recommends tracks based on a user's listening time, number of clicks, collection, and download behaviour. The music recommendation system's data content primarily consists of user data, music data, and user-system interaction behaviour data. Basic information about the user is contained in user data. Music data contain various details about music and can be used to extract interesting features, making it an important data source for recommender systems. The user's interaction with music is included in user behaviour data, and the recommendation system can be used to mine the user's potential information. The purpose of data processing technology is to clean, process, and transform the system's data so that the algorithm layer can obtain clean and effective data, thereby improving the recommendation system's performance. The validity of the behaviour data directly affects whether the recommendation result can meet the user's needs because the user's historical behaviour information reflects the user's preferences at different times. The background log information will record each user's behaviour, such as clicking on music, commenting on music, and sharing music, and the stored content format will be in the form of a dictionary. Finally, a data format that is beneficial to the calculation of the recommendation algorithm can be obtained after systematic processing. The information gathered will be processed. Missing data, data noise, and data duplication may occur during the data collection and transmission process, affecting subsequent model training and resulting in low model robustness. As a result, the information must be processed. There may be many data attributes when analyzing and processing data, but some are irrelevant and some are relevant, so it is necessary to select the most relevant features for processing to improve the model's robustness. The accuracy of a recommendation is insufficient. The diversity of recommendation results is critical with the growing number of Internet services and changing user needs. If users listen to ancient songs for a long time, for example, our recommendation list should include some variety based on personalization and precision, such as sad songs that are not very similar to ancient styles. The recommendation is successful if the user clicks. The recommendation results differ depending on each user's unique historical behaviour data. The system can update the recommendation in real time based on short-term data and long-term data, allowing the user to experience the system's personalization. The recommender system learns from the user's past behaviour and improves its personalization and accuracy over time.

The higher the big data recommendation model's evaluation value, the more interested in music the user is; the big data recommendation model is generated into the nearest neighbour set, which is the user's big data recommendation model set that is similar to the user's interest. Two user big data recommendation models are regarded as two vectors in the vector space using the method of vector space similarity calculation, and the similarity between them is measured by calculating the cosine value of the angle between the two vectors in the big data recommendation model. Finally, the big data recommendation model's recommendation set is generated. The user's evaluation value of the song is predicted based on the similarity between neighbour users and the user as well as the neighbour users' evaluation value of the song. Then, using the big data recommendation model, the first few songs with the highest ratings are measured, and the recommendation results are fed to the model's first few users. To begin, their features are extracted to generate the user interest model of the big data recommendation model based on the music resources downloaded, searched, and rated within a certain period of time according to the big data recommendation model, and then different big data recommendation models are generated from the ringtone resources in the ringtone library. The content recommendation set is made up of music and user interest models with similar attribute values; second, the big data recommendation model predicts the user's predicted score for some songs and finds the nearest neighbour based on the users with similar interests. The big data recommendation model's recommendation set is recommended; third, the content recommendation set in the recommendation set and the music sorted by the nearest neighbour big data recommendation model are scored according to the weight, and the big data recommendation model with the highest score is chosen as the final recommendation item to be recommended to the user.

## 5. Experiments on Proposal Models Based on Big Data

The individualization music proposal model of big data technology proposed in this study introduces the GRU network after the XCNN network, which has long-term memory ability and can extract the feature relationship between pre- and post-sequence images. In order to verify the music classification effect of the CURNN model in this study, the experimental results are compared with music classification methods such as HCRNN, FCN6, and DielemanCNN, and the accuracy, AUC, and mean average accuracy mAP of each method are calculated. The results are shown in Figure 4.

It can be seen from the experimental data that CURNN has higher accuracy, AUC, and mean average accuracy rate mAP than the other three models due to the addition of a big data proposal model. The closer the accuracy, AUC, and mAP values are to 1, the better the classification effect is, so the classification effect of the model CURNN proposed in this study is much higher than that of DielemanCNN and FCN6 that only use their own data. Compared with the HCRNN model that also uses the RNN network, CURNN is still ahead. For the three music proposal models proposed in this article, the user's score is predicted on the collection of songs; the predicted scores of 10 to 100 songs are randomly selected; and the *L*, *R*, and *G* values are calculated. The experimental results are shown in Figures 5–7.

As the number of predicted scores increases, the parameter scores decrease continuously. According to the experimental results, the prediction scores of the prediction results of the big data proposal model are higher than those of the other two models, and it has a better proposal effect. The user's behaviour is temporal, so time weights should be introduced into the user prediction scoring formula. Different time weights have different effects, thus affecting the final proposal result. This study sets the time weight value of 0.1 to 0.9 for comparative experiments. In this section, the experimental results will be displayed and analyzed, and the evaluation indicators will be precision rate, recall rate, and *F*1 score. The specific experimental results are shown in Figures 8–10.

The relationship between the time weight coefficient, precision rate, recall rate, and *F*1 is neither positive nor negative, as can be seen. Precision, recall, and *F*1 scores increase steadily as the time weight increases, and when the time weight reaches 0.4, the three indicators' scores tend to be flat. To summarize, the proposed big data music proposal model is about 20% more accurate than the collaborative filtering model and the hybrid model when the time weight is 0.4. And the big data-based proposal algorithm is clearly superior to the single similarity proposal algorithm.

## 6. Conclusions

Traditional proposal methods frequently limit themselves to user behaviour data while ignoring background data and other issues. This study investigates a data collection method that combines system logs, system databases, network interfaces, and sensors; collects data from multiple sources; and prepares a complete data set for individualization proposals, in conjunction with the big data collection method. Following the completion of data collection, this study uses the appropriate standardization processing methods to perform data standardization work in the preprocessing according to the various types of data collected. We start with two aspects in the proposal candidate set screening stage. On the one hand, it seeks out similar users' favorite music, and on the other, it uses clustering to find music that is similar to the user's favorite music. Starting with two aspects, it ensures that the candidate set is personalized, as well as fully covering the user's interests and improving the quality of the final proposal results. Massive music works and users cause a slew of issues for recommender systems. This study solves the problem of cold start and hot item processing by increasing proposal probability and decreasing item weight, which not only improves the coverage of the proposal system but also ensures the accuracy of the proposal, thus alleviating these issues. The ability of the system to process data is also important in the big data environment. Using the Hadoop big data processing framework, this study improves the system's processing ability. To begin, the recommender system's functional and nonfunctional requirements are analyzed, and various designs required for system implementation are completed. A working environment is created in which a music individualization proposal system can be implemented. Finally, testing is used to confirm the system's feasibility and effectiveness. To mine user preferences and complete the recommendation process, this study primarily uses user data, music work data, user behaviour data, and behaviour context data. However, there is a lot of data that can be added to the recommendation process calculation. Tag data are typically used by users to mark their feelings and experiences with musical works, allowing tags to link users to musical works. These data should be the focus of future research.

## Figures and Tables

**Figure 1:** Proposal process based on big data technology.

**Figure 2:** The interactive ritual chain linked to emotion in music.

**Figure 3:** Big data music individualization proposal process.

**Figure 4:** Comparison of different model experiments.

**Figure 5:** Comparison experiment of *L* value of different models.

**Figure 6:** Comparison experiment of *R* value of different models.

**Figure 7:** Comparison experiment of *G* values of different models.

**Figure 8:** Improved big data proposal model.

**Figure 9:** Improved collaborative filtering proposal model.

**Figure 10:** Improved hybrid proposal model.

## Data Availability

The data used to support the findings of this study are available from the corresponding author upon request.
